The article "Recent Advances in Thermally Activated Delayed Fluorescent Polymer—Molecular Designing Strategies" was published in 2020. Journal: Front Chem.

# Recent Advances in Thermally Activated Delayed Fluorescent Polymer—Molecular Designing Strategies

**DOI:** 10.3389/fchem.2020.00725

**Published:** 2020-08-14

**Authors:** Xia Yin, Ying He, Xu Wang, Zexin Wu, Erbao Pang, Jing Xu, Jun-an Wang

**Affiliations:** ^1^Department of Polymer Materials, School of Materials Science and Engineering, Shanghai University, Shanghai, China; ^2^Institute of Materials, School of Materials Science and Engineering, Shanghai University, Shanghai, China

**Keywords:** organic light-emitting diodes, thermally activated delayed fluorescence, electroluminescence, TADF polymer, quantum efficiency, molecule designing

## Abstract

Thermally activated delayed fluorescent (TADF) materials, as the third generation of organic electroluminescent materials, have many advantages over other organic light-emitting diodes (OLEDs) materials, such as 100% internal quantum efficiency, no doping of heavy metals, and avoiding the shortages of ordinary fluorescent materials and phosphorescent materials. So it is considered to be the most competitive organic light-emitting materials, and has great application prospects in the field of OLEDs. So far, small-molecule TADF materials have achieved high quantum yield and full-color range of red, green, and blue. However, TADF polymers suitable for low-cost and easily scalable solution processing are less developed, which are confined by the preparation methods and polymers designing, and there are still challenges of increasing quantum efficiency and strengthening device performance. This review mainly summarizes different synthesis strategies of TADF polymers and the latest development in the field. Special attention is focused on illustrating the designing and structure-property relationship of TADF polymers, and finally, an outlook is given for the design and application prospect of TADF polymers in the future.

## Introduction

OLEDs are high-brightness, wide-view, and fully cured light emitting devices. As OLEDs have the advantages of low driving voltage, fast response speed, high luminous efficiency, simple manufacturing process and easy panchromatic display, they are considered as “Fantastic display,” and one of the most important flat-panel display technologies in the future (Sheats et al., 1996). The classical three-layer OLED device structure is composed of an electron transport layer (ETL), a hole transport layer (HTL), and an emitting layer (EML) (Wang et al., 1999). Among them, the emitting layer material not only largely determines the performance of the device, but also has a great influence on the processing method of the device. It is currently one of the most promising materials to improve the device performance.

The article "Recent Advances in Thermally Activated Delayed Fluorescent Polymer—Molecular Designing Strategies" was published in 2020. Journal: Front Chem.

At present, the mainstream luminescent materials used in the emitting layer include traditional fluorescent materials, phosphorescent materials, thermally activated delayed fluorescent materials, etc. (Köhler et al., 2002; Xiao et al., 2014). In fluorescent materials, the luminescence is accomplished by exciton transition from singlet state to ground state (Pope et al., 1963; Rothberg and Lovinger, 1996), while the luminescence of phosphorescent materials comes from exciton transition from triplet state to ground state (Baldo et al., 1998). Thermally activated delayed fluorescent (TADF) materials have a totally different luminescence mechanism, in which the exciton transition from triplet excited state to singlet excited state occurred through reverse inter-system crossing (RISC), thereby transition radiative emission (Nakagawa et al., 2012; Tanaka et al., 2012; Uoyama et al., 2012). Although those materials have different luminescence mechanisms, the structure and working principle are similar when they are used as emitting layer in OLED devices.

The performance of luminescent materials directly affects the luminous efficiency of the device. Therefore, a lot of researches on OLEDs are focused on the behavior of luminescent materials, including the electroluminescence (EL) efficiency, radiative lifetime and color purity. Meanwhile, a variety of matching auxiliary materials, such as hole transport materials, electron transport materials, exciton blocking materials and host materials, have been researched and developed to maximize the performance of the luminescent materials, and thereby to obtain OLED devices with excellent performance. In the past three decades, OLEDs have been well commercialized due to the maturity of fluorescent and phosphorescent materials. However, both fluorescent and phosphorescent materials still have fatal defects. The maximum device internal quantum efficiency (IQE) of conventional fluorescent materials is confined to within 25%, due to the low singlet excitons generation ratio of 25% in device. The luminescence of phosphorescent materials was improved by strengthened spin-orbit coupling (SOC) via doping heavy metals such as iridium (Ir) and platinum (Pt), while those materials also have uncertain toxicity, high cost and limited emission in blue regions (Holmes et al., 2003; Zhang et al., 2014b), etc. Promisingly, thermally activated delayed fluorescence supplies a solution to utilize triplet excitons emission by RISC process, where triplet excitons can be effectively upconverted into singlet state and decayed via a radiative channel to the ground state. Theoretically speaking, TADF-OLEDs may reach 100% IQE under EL operation.

The article "Recent Advances in Thermally Activated Delayed Fluorescent Polymer—Molecular Designing Strategies" was published in 2020. Journal: Front Chem.

As early as 1961, Parker and Hatchard (1961) discovered the TADF phenomenon in the magenta dye, and subsequently observed the same phenomenon in fullerenes and other compounds under photoexcitation. In 2009, Adachi et al. (Endo et al., 2009) introduced TADF materials into OLED devices for the first time. Since then, TADF materials have made great progress in OLED applications, but the most interested TADF emitters so far are small molecules, due to the ease in simultaneously achieving a small singlet-triplet energy splitting (Δ*E*_ST_) and suppressing the internal conversion (IC) process of the molecule. TADF polymers have excellent modifiability and good thermal stability compared to small molecules. More importantly, narrow band-gap TADF polymers with robust, high film-forming property have emerged, which is extremely beneficial for simple roll-to-roll printing (Wang et al., 2020). In addition, compared with small molecules, self-host TADF polymers are more likely to be prepared by rational group modification and structure regulation to solve the phase separation problem of host-guest-doped TADF-OLEDs. Due to those process-related problems, research and development are shifting to TADF polymers. The existing research strategies of TADF polymers are mainly on indirect synthesis, in which the active unit with TADF emission was embedded or grafted into the polymer as a main chain (Nikolaenko et al., 2015; Lee et al., 2016), side chain (Luo et al., 2016) or dendrimer core (Albrecht et al., 2015). Those previous research results bring significant clues for designing and synthesis of new TADF polymers. This review firstly introduces the luminescence mechanism of TADF materials, and briefly analyzes the design principles of TADF materials, focusing on the existing TADF polymers. Finally, the future development of TADF materials is prospected from the aspects of material synthesis, performance and application.

## Luminescence Mechanism of TADF Materials

The OLED device is generally composed of an anode, a metal cathode and organic function layers. According to the number of organic function layers, OLED devices can be classified into single-layer structure, double-layer structure, three-layer structure and multilayer structure. Three-layer device structure is most commonly used in organic light-emitting device (Adachi et al., 1988; Dai et al., 2005). This structure is mainly composed of ETL, HTL and organic EML, which is not only conducive to selecting materials as functional layers but also to optimizing device performance.

Under the action of external voltage, holes and electrons are injected from the anode and the cathode respectively, passing through the respective transport layers and finally combing to form excitons in the light-emitting layer (Hung and Chen, 2002). Those excitons contain both singlet excitons (S_1_) and triplet excitons (T_1_) due to their different spin states before and after excitation, and the ratio of S_1_ to T_1_ is 1:3 according to the spin quantum theory (Rothberg and Lovinger, 1996). Emission comes from the radiative transition of the exciton, that is, from singlet or triplet state to the ground state. During this process, photons generate and emit out from the EML which results in different efficiencies of OLED devices.

The article "Recent Advances in Thermally Activated Delayed Fluorescent Polymer—Molecular Designing Strategies" was published in 2020. Journal: Front Chem.

As shown in Figure 1, unlike conventional fluorescence and phosphorescence in OLEDs, TADF emission has two distinct components: prompt fluorescence (PF) and delayed fluorescence (DF). Since the energy levels of the S_1_ state and the T_1_ state of the TADF molecules are close to each other (Δ*E*_ST_ < 0.5 eV), it is possible to use heat in the environment to achieve the reverse inter-system crossing (T_1_ → *S*_1_), thereby converting the triplet excitons, accounting for 75% of total excitons, into singlet excitons, and the radiative transition produces delayed fluorescence of microsecond or even millisecond lifetime. On the other hand, the rapid radiative transition of excitons originally occupied in the S_1_ state, accounting for 25%, produces nanosecond-order prompt fluorescence. Thus, theoretically, TADF molecule could achieve 100% internal quantum efficiency. Since both PF and DF are derived from singlet state emission, they are completely identical in the emission spectrum.

**Figure 1:** Luminescence mechanism of TADF. F, P, PF, DF, TADF, IC, ISC, RISC and Δ*E*_ST_ denote fluorescence, phosphorescence, prompt fluorescence, delayed fluorescence, thermally activated delayed fluorescence, internal conversion, inter-system crossing, reverse inter-system crossing and singlet—triplet state energy splitting, respectively.

The TADF emission process is based on the spatial separation of the highest occupied molecular orbit/the lowest unoccupied molecular orbit (HOMO/LUMO) of charge transfer (CT) excited state materials (Peng et al., 2013). The energy levels between the lowest singlet state and the lowest triplet state are close due to weak electron exchange, thus Δ*E*_ST_ is very small in TADF molecules. It is easy to achieve the reverse inter-system crossing under the thermal activation condition, thereby converting the triplet excitons into singlet excitons and accomplishing 100% internal quantum efficiency.

## TADF Molecular Structure Design

### Design Principle of TADF Molecule

Although TADF has a unique RISC process and its mechanism is complex, the design of TADF materials has certain rules. In the case of TADF organic small molecules, HOMO is usually located on the electron donor (D), and LUMO on the electron acceptor (A). For this reason, groups with greater steric hindrance (Mehes et al., 2012; Zhang et al., 2012; Kawasumi et al., 2015; Suzuki et al., 2015; Feuillastre et al., 2016; Furue et al., 2016) were generally introduced between the donor and the acceptor of the molecules, for obtaining spatial separation of HOMO and LUMO to enhance the charge transfer state (Xie and Li, 2017). From the perspective of molecular design strategy, TADF polymer draws on the design idea of the electron donor-electron acceptor (D-A) structure of the TADF organic small molecules, that is, the electron donor and the acceptor units are connected in a specific way in the polymer (Zhang et al., 2014a; Numata et al., 2015; Suzuki et al., 2015). By regulating the interaction between the electron donor and the acceptor and the degree of electron cloud overlap to reduce Δ*E*_ST_, the reverse inter-system crossing process will be enhanced to achieve the TADF effect (Endo et al., 2011; Lee et al., 2012). However, combined with photoluminescence quantum yield (PLQY) that is one of the important properties when TADF polymer is used as an emissive layer in OLEDs, a certain degree of spatial overlap between HOMO and LUMO is a necessary according to Franck-Condon theory. So, when regulating the degree of spatial separation of HOMO/LUMO to achieve small Δ*E*_ST_ in TADF polymers, the degree of spatial overlap between them should be considered to ensure a relatively high PLQY. For this, the TADF polymer should possess a rigid structure to reduce the recombination energy of the molecule, thereby suppressing non-radiative transitions to obtain a higher rate of radiation decay (Guo et al., 2017).

The article "Recent Advances in Thermally Activated Delayed Fluorescent Polymer—Molecular Designing Strategies" was published in 2020. Journal: Front Chem.

However, compared with small molecules, in TADF polymers, triplet excitons are more prone to quenching due to triplet—triplet annihilation effect (TTA) within and between molecules, and it is a dilemma to obtain a smaller Δ*E*_ST_ and to inhibit non-radiative internal conversion in polymers containing a large number of atoms. In addition, due to the through-bond charge transfer effect of the conjugated structure, the emission wavelength of TADF polymer will show a large red shift, leading to the majority of TADF polymer emission concentrated in orange and green light emission, which is unfavorable for achieving blue light emission of TADF polymer. TADF polymer light-emitting diodes (PLEDs) have also been reported to have serious efficiency roll-offs and low external quantum yield (EQE) till now. To address these issues, TADF polymer design strategies are particularly of significance (Liu et al., 2018a).

### Common Electron Donor and Electron Acceptor Units

In the design of TADF polymers, it is extremely important to select the appropriate functional group. It has been reported that a large number of functional groups, such as electron donor and acceptor groups, are connected to each other in a specific manner to achieve the TADF effect. Presently, the electron donor of D-A type TADF polymer is mainly composed of N-containing aromatic groups with strong electron donating ability, which requires high triplet energy level, good stability, and excellent carrier transport capacity. Common electron donors include carbazole, phenoxazine, aniline, acridine and their derivatives. For electron acceptors, there are mainly the following types: nitrogen heterocycles, benzophenones, cyanobenzenes, diphenylsulfones and their derivatives, etc. (Volz, 2016), which generally have strong electron-withdrawing ability and good electron-conjugation properties, and a molecular structure to be easily modified.

## TADF Polymer

Although most of the TADF materials are usually small organic molecules due to a direct design for their electronic structures, the processing is expensive and cannot be used for large device fabrication. Compared with small molecules, polymers are extremely suitable for solution processing, such as spin coating, inkjet printing, and roll-to-roll coatings (Gustafsson et al., 1992; Wu et al., 2009), showing a great potential in low-cost processing and large-scale applications. At present, the main design strategy of TADF polymer is based on an indirect way that introduces small molecules with known TADF-active behavior into different positions of the polymer structure either as pendant groups, as main chain constituents, or as core. Beside of these, there are also self-emission TADF polymers. In this case, small molecules that originally do not have TADF properties reduce the energy splitting between corresponding ^1, 3^CT after polymerization due to the expansion of the conjugated structure, making Δ*E*_ST_ relatively small enough to be overcome by heat, so the polymer shows excellent TADF properties (Wei et al., 2017).

Therefore, in this section, TADF polymers are classified as according to the position of TADF active units in the polymer structure, as shown in Figure 2: (1) Core-acceptor / Shell-donor dendritic TADF polymer; (2) Main chain TADF polymer; (3) Backbone-donor/Pendant-acceptor TADF polymer; (4) Side chain TADF polymer; (5) Self-emission TADF polymer. Each type is further subdivided on the basis of the connection mode of its electron acceptor and electron donor. For example, dendritic TADF polymers have conjugated and non-conjugated structures depending on the linking groups of the core and the acceptor. Based on the molecular structure of TADF fragments on the backbone, the main chain TADF polymer can be divided into D-A type TADF polymer with alternating copolymerization of donor and acceptor and B-T-B type TADF polymer with spaced backbone. The side chain TADF polymers are classified into conjugated and non-conjugated in the light of the difference of the backbone structure. According to the connection mode of the electron donor and the acceptor in the TADF fragment, the side chain non-conjugated TADF polymer is divided into D-A directly connected intramolecular charge transfer polymer and space charge transfer polymer where donors and acceptors are separated. It is found that the conjugation effect, TADF fragment structure, and D-A connection mode affected the properties of TADF polymer emitters, such as the charge carrier mobility, emission color, and efficiency of TADF properties.

The article "Recent Advances in Thermally Activated Delayed Fluorescent Polymer—Molecular Designing Strategies" was published in 2020. Journal: Front Chem.

**Figure 2:** TADF polymer design strategy. **Type 1:** TADF dendrimer with the acceptor as the central core and the peripheral donor as the dendrons. **Type 2:** TADF polymer with completely alternating connection of donor and acceptor (upper); TADF moieties separated by backbone spacer units (lower). **Type 3:** Donors fixed as backbone and acceptors grafted on the side-chain. B, D, P and A denote backbone, donor, pendant and acceptor. **Type 4:** TADF moieties embedded into backbone as a pendant (upper); donor and acceptor molecularly separated while spatially close (lower). **Type 5:** The whole polymer exhibiting TADF effect rather than the small molecule monomer.

### High Molecular Weight TADF Dendrimer

Dendrimer (Astruc et al., 2010) is a perfectly branched polymer with precise molecular structure, usually a core-shell structure consisting of a central core and a repeating branch perimeter. Dendritic TADF macromolecules have both the advantage of high molecular weight similar to polymers and the same precise molecular structure as small molecules, so the required photoelectric and processing properties of the materials can be enhanced by regulating the molecular structure (Burn et al., 2007). Meanwhile, owing to their unique structure with a high steric hindrance, they are generally in a soluble and amorphous state, and can isolate chromophores at the core to prevent concentration quenching. Thus, dendritic TADF macromolecules are ideal for solution-processing in OLED devices.

Currently, TADF dendrimer has been widely studied and applied to OLED devices with excellent performance. The central core of a dendritic TADF polymer is the main unit contributing to the TADF performance. Usually, the structure of the central core, mostly D-A type structure, is similar to that of small molecule TADF units. Common electron acceptor units such as dibenzophenone, triazine and diphenylsulfone are often used as the core of the acceptor. Depending on the functional groups connecting the core and peripheral dendrons, TADF dendrimers often have conjugated and non-conjugated structures. On account of the strong molecular rigidity in the conjugated structure, the solubility of the molecule will be reduced, and the expanded conjugation on the periphery will interfere with the emission of the core, causing the emission color to change. Flexible alkyl chains (Xu et al., 2008) are often chosen to enhance molecular solubility, facilitate charge transfer, and encapsulate the luminous core.

The article "Recent Advances in Thermally Activated Delayed Fluorescent Polymer—Molecular Designing Strategies" was published in 2020. Journal: Front Chem.

Triazine and its derivatives have strong electron-withdrawing ability and excellent structural modifiability, so they are fairly good acceptor cores. Through modification of dendritic donor substituents, TADF dendrimers can be effectively constructed.

Yamamato's team (Albrecht et al., 2015) has attempted a series of carbazole dendritic macromolecules (GnTAZ) with triphenyl-s-triazine nuclei, and successfully achieved a solution-processable non-doped high molecular weight TADF dendrimer. In their work, the singlet-triplet state energy splitting of the molecules was determined by fluorescence and phosphorescence spectroscopy measurements, and the Δ*E*_ST_ was calculated to be 0.03, 0.06, and 0.06 eV for G2TAZ, G3TAZ, and G4TAZ, respectively, which is sufficiently low to allow inverse inter-system crossing from triplet state to singlet state at room temperature. Due to the intense overlap of HOMO and LUMO orbitals, G1TAZ exhibits non-TADF properties, while other dendrimers possess thermally activated delayed fluorescence. The pure spin-coated films of the GnTAZ (*n* = 2,3,4) dendritic polymers also show TADF emission with a moderate PLQY, and a maximum EQE of 3.4% (G3TAZ) is acquired on the OLED devices fabricated with those polymers as the light-emitting layer.

Besides, Yang et al. (Li et al., 2016) proposed a strategy for preparing TADF emitters for solution process, i.e., polycarbazole encapsulation. They developed a green-emitting TADF core (DMAC-BP) and synthesized two TADF dendrimers (CDE1 and CDE2, exemplified in Figure 3). Both dendrimers had excellent thermal stability, good solution processability and significant TADF characteristics. For example, with CDE1 dendrimer as emission layer, a non-doped OLED prepared by solution process shows a high EQE of 13.8%, demonstrating a complete harvest of all the excitons generated by the two parallel emission channels of TADF and the exciplex emission. It is worth noting that the EQE of the dendrimers was still as high as 13.3% even at the high brightness of 1,000 cd·m^−2^. This work, by combining the two parallel emissive channels, provided a novel and efficient design strategy for non-doped solution-processed TADF emitters.

The article "Recent Advances in Thermally Activated Delayed Fluorescent Polymer—Molecular Designing Strategies" was published in 2020. Journal: Front Chem.

**Figure 3:** Chemical structures of DMAC-BP, CDE1, and CDE2.

Sun et al. (2018) designed and synthesized two new dendrimers (G-TCTA and G-mCP, see Figure 4), which had effective non-conjugated connections between TADF core (G-G0) and different excited complex dendrites. The dendrimer G-mCP exhibited a smaller Δ*E*_ST_ (0.08 eV) and a higher PLQY (90%). As the photophysical properties of the TADF core and the function of exciplex in the dendrimer are independent as a result of the non-conjugated linkage, the solution-processed G-mCP non-doped device achieved a very low drive voltage of 2.7 V and a high power efficiency of 46.6 lm·W^−1^ with a maximum EQE up to 16.5%.

**Figure 4:** Chemical structure of G-G0 and its dendritic derivatives G-mCP and G-TCTA.

The aggregation-caused quenching effect (ACQ) makes the material in the aggregated state weaken in fluorescence or even emit no fluorescence, which seriously affects the practical application of luminescent materials. To overcome this problem, through combination of aggregation-induced delayed fluorescence (AIDF) effect and a strategy of aggregation-induced emission (AIE) molecular design, Wang et al. (2019b) developed TADF dendrimer which effectively improved the efficiency roll-off in solution-processed OLEDs.

Shao and Wang's group reported the design of spatial charge transfer hexaarylbenzenes (TSCT-HABs) containing circularly arranged electron donors (acridines/dendritic triacridines) and acceptors (triazines), as shown in Figure 5. In TSCT-HABs, the spatial p–p interaction between the donor and acceptor provided efficient full space charge transfer emission, and the spatial separation of donor and acceptor caused a Δ*E*_ST_ of 0.04–0.08 eV, resulting in a delayed fluorescence (microsecond order). The results indicated that these propeller-like structured dendrimers exhibited TADF and AIE effects in OLEDs prepared by solution processing. The emission intensity of these dendrimers from the solution to the aggregated state is increased by 6–17 times. TSCT-HABs-based solid solution OLEDs had a maximum EQE of 14.2%, making them one of the most efficient emitters of solid solution TADF OLEDs.

**Figure 5:** Chemical structure of space charge transfer TADF dendrimer TSCT-HABs.

Using the traditional design principle of molecular charge transfer, Wang et al. (2019a) designed and synthesized two dendrimers CzTAZPO and sCzTAZPO with AIE and TADF characteristics, as shown in Figure 6. Both molecules had asymmetric D-π-A configurations, in which triazine was used as the electron acceptor, the carbazole dendrimer as the electron donor, and the phenyl spacer as the π-bridge, forming a highly distorted conformation between a carbazole dendrimer and a phenyl spacer. In addition, a phosphorus oxy group was added to improve the electron transport performance. Theoretical calculations and experimental results showed that the increase in the number of carbazole dendrites led to an increase in the intensity of the fluorescent oscillator, while the Δ*E*_ST_ value decreased. CzTAZPO and sCzTAZPO showed significant AIE and TADF characteristics, and CzTAZPO-based non-doped OLEDs showed high efficiency (EQE_max_ = 12.8%) and low efficiency roll-off (<1.6%).

The article "Recent Advances in Thermally Activated Delayed Fluorescent Polymer—Molecular Designing Strategies" was published in 2020. Journal: Front Chem.

**Figure 6:** Chemical structures of CzTAZPO and sCzTAZPO.

### Main Chain TADF Type Polymers

The design strategy of the main chain type TADF polymer is to connect the small molecule TADF unit into the main chain of the polymer by chemical bonding, wherein the electron donor and the electron acceptor can be completely and alternately connected (alternating D-A type) as the TADF unit to construct polymer backbone. A conjugated or non-conjugated functional unit might as well be introduced as a spacer group into the polymer backbone (interval B-T-B type) to modulate the photoelectric properties of the TADF polymer.

#### Alternating D-A Type

In some TADF polymers, the electron donor and the acceptor are alternately connected as a TADF light-emitting unit, thus forming the backbone of the polymer. These polymers generally have a planar conjugated characteristic, which is advantageous for expanding the degree of conjugation and achieving high carrier transport performance, and a large rigid structure which is conducive to improving the radiation decay rate, thereby increasing the quantum luminescence yield (Zhang and Cheng, 2019). However, there is inevitable non-radiative transition inducing excitons dissipation due to potential conjugation and interactions between D/A units. On the other hand, the rigid configuration of the molecules makes the twist between D and A difficult, which results in the HOMO/LUMO still overlap spatially to a certain extent.

Adachi group (Lee et al., 2016) reported two D-A type π-conjugated TADF polymers (pCzBP and pAcBP) whose backbones were composed of electron donor carbazole or an acridine group and electron acceptor diphenyl alternately for the first time. The synthesized TADF polymers exhibited smaller Δ*E*_ST_ (0.18 and 0.10 eV). Theoretical calculations showed that the HOMO was mainly located in the electron donor unit, carbazole or acridine, and the LUMO mainly in the electron acceptor unit, benzophenone. Experiments that the delayed emission intensity with the microsecond lifetime decreased when the temperature dropped from 300 to 50 K, confirm the TADF characteristics of the polymers. The green emitting OLEDs had EQE of 8.1% (pCzBP) and 9.3% (pAcBP), respectively, and the EQE remained as high as 8.0% even at a high luminance of 1,000 cd·m^−2^.

The article "Recent Advances in Thermally Activated Delayed Fluorescent Polymer—Molecular Designing Strategies" was published in 2020. Journal: Front Chem.

Huang et al. (Hu et al., 2018) reported a main-chain blue TADF polymer (P0, Figure 7), which was alternately connected by electron-deficient diphenylsulfone and electron-rich trianiline. The doped OLED device prepared by solution treatment of P0-based TADF polymer exhibited pure blue emission with a Commission Internationale de l'Eclairage (CIE) coordinate of (0.16, 0.10) and a maximum EQE of 5.3%. In their work, a series of color-tunable polymers had also been developed by incorporating triphenylamine functionalized triazine group, a narrow bandgap unit which could control the emission color of the polymer. These polymers exhibited delayed fluorescence and emitted light from sky-blue to blue-green, and the luminous efficiency was significantly improved. It has been demonstrated that a blue-green PLED based on polymer P3 possesses a maximum EQE of 8.7%.

**Figure 7:** Chemical structure of PTSn (*n* = 0–5).

#### Interval B-T-B Type

Organic electroluminescent devices based on TADF luminescent molecules often have serious efficiency roll-off problems during service, which is mainly due to the concentration quenching caused by the long lifetime of triplet excitons. For this case, the molecular excited states have microsecond life, which leads to the increase of exciton concentration and formation of “hot” exciton that destroys the chemical bonds of the luminescent molecules, finally resulting in a decay process of the device (Cai and Su, 2018). Therefore, the designing strategy should concentrate on introduction of the backbone spacer group to prevent the aggregation of the TADF emitter center. This spacer group should have a certain steric hindrance, reduce the conjugation degree of the main chain, improve the triplet energy level of the main chain, and avoid the quenching of the triplet excitons. In the interval B-T-B type TADF polymer, a conjugated or non-conjugated functional unit as a spacer group is introduced, so the emitter centers on the main chain are separated from each other, without forming a conjugated system, thus possibly regulating the photoelectric properties of TADF polymer.

The article "Recent Advances in Thermally Activated Delayed Fluorescent Polymer—Molecular Designing Strategies" was published in 2020. Journal: Front Chem.

In 2015, Nikolaenko et al. (2015) proposed a strategy called “intermonomer TADF,” in which TADF active units were indirectly prepared from the polymerization of donor and acceptor monomers. During the polymerization process, the monomeric CT emitter was formed from the donor triphenylamine and the acceptor triphenyltriazine monomer, which could serve as charge transport units. And a host material with a high triplet energy level, 2,2',5,5'-tetraethyl-1,4-diphenylbutane, was connected to the main chain as a spacer unit to co-construct a TADF emitter polymer as shown in Figure 8. This molecule construction not only effectively avoided the aggregation of TADF active center, but also inhibited the quenching problem caused by aggregation and triplet-triplet annihilation. Furthermore, it greatly improved the solubility of the polymer, which was beneficial to the preparation of solution processable OLED. A non-doped OLED device prepared by solution method, in which the synthesized intermonomer TADF polymer acted as emitting layer, emitted in a green region, having a maximum EQE up to 10%, and a CIE coordinate of (0.32, 0.58).

**Figure 8:** TADF polymer structure for intermonomer strategy.

Liu et al. (2019) reported new conjugated and non-conjugated interval B-T-B type TADF polymers, which effectively reduced the steric resistance of the spacer element, avoided the quenching of the triplet excitons, and significantly improved EQE with low efficiency roll-off.

The research group directly embedded the small molecule blue TADF emitter (BOPAC-TRZ) into the poly (arylether) (PAE) backbone to synthesize the blue TADF polymer, as shown in Figure 9. In this polymer, the oxygen atoms could not only interrupt the conjugation to maintain the high *E*_T_ of the polymer backbone, but also inhibit electron transport between adjacent TADF fragments to avoid red shift. Since the oxygen-induced electron transport among adjacent TADF units was negligible, the corresponding blue delayed fluorescence property of the TADF small molecule could be inherited by the synthesized polymer. Through device optimization, the efficiency of the PLED based on P(BOPACTRZ-BPA) reaches 29.7 cd/A (21.2 lm/W, 13.2%) with a small roll-off, and the CIE coordinate is (0.18, 0.32). Recently, the team (Rao et al., 2020) made breakthroughs in conjugated TADF polymers. They designed a variety of methyl substituted phenylene linking units as backbone spacer groups, and through polymerization of these groups with D-A-D TADF fragments (AcBPCz), successively synthesized a series of TADF conjugated polymers, Poly(AcBPCz-P), Poly(AcBPCz-DMP), and Poly(AcBPCz-TMP), as shown in Figure 9. Interestingly, they found that with the increase of the number of methyl substituents on the phenylene group, the Δ*E*_ST_ of the polymer gradually decreased, and the TADF emission gradually enhanced. The experiments show that the conjugated polymer Poly(AcBPCz-TMP) having tetramethyl-substituted phenylene group as linking unit exhibited almost the same TADF effect and excellent electroluminescence properties as the TADF emissive small molecule AcBPCz. The corresponding solution-processed monochromatic OLED device exhibited blue-green emission with a wavelength of 507 nm and a maximum EQE of 23.5% (68.8 cd/A, 60.0 lm/W). By mixing orange-red light TADF emitter NAI-DMAC into the Poly(AcBPCz-TMP) luminescent layer, a warm white optical device was prepared, in which the CIE coordinate was (0.36, 0.51), and the maximum EQE reached 20.9% (61.1 cd/A, 56.4 lm/W).

The article "Recent Advances in Thermally Activated Delayed Fluorescent Polymer—Molecular Designing Strategies" was published in 2020. Journal: Front Chem.

**Figure 9:** Chemical structure of TADF polymers, P (BOPACTRZ-B), P (BOPACTRZ-BPA), Poly (AcBPCz-P), Poly (AcBPCz-DMP) and Poly (AcBPCz-TMP).

### Backbone-Donor/Pendant-Acceptor Type TADF Polymers

In the above strategy, the electron donor and the electron acceptor are alternately arranged in the main chain backbone. The alternating D-A conjugated polymer is mostly of a planar geometric feature, which is advantageous for expanding the conjugation and achieving high charge transfer, and the rigid configuration is favorable for high rate of radiation decay so as to obtain high PL quantum yield. However, this results in an inevitable large spatial overlap of the HOMO/LUMO of the donor and acceptor. In this case, the polymer generally requires higher exchange energy, while the latter greatly limits the lowering of singlet—triplet energy splitting [Δ*E*_ST_ close to 0.7 eV (Köhler and Bässler, 2009)], and thus is not conducive to obtaining an effective TADF effect.

It has been proved theoretically and experimentally (Tao et al., 2014) that highly efficient D-A-linked pure organic TADF molecules mostly require an almost orthogonal structure of the donor and acceptor to reduce the HOMO/LUMO overlap of each other. However, as Figure 10 shows, the D-A orthogonal configuration of TADF polymer usually has large steric hindrance, so it is difficult to synthesize D-A orthogonal structure in the main chain backbone. Whereas, in the TADF polymer designed by the Backbone-donor/ Pendant-acceptor (BDPA) strategy, the electron donor unit is fixed on the backbone of the conjugated polymer, and the electron acceptor is grafted on the side chain orthogonally. The donor is delocalized throughout the polymer backbone so that it has a conjugated property to ensure more efficient charge injection and transfer characteristics. In addition, there is a certain twist between the D-A, which is beneficial to the further separation of the molecular frontier orbitals to obtain a very small Δ*E*_ST_. This twisted D-A structure can be retained along the suspension direction in the polymer to ensure the TADF emission characteristics and achieve high efficiency of delayed fluorescence.

The article "Recent Advances in Thermally Activated Delayed Fluorescent Polymer—Molecular Designing Strategies" was published in 2020. Journal: Front Chem.

**Figure 10:** Difference between planar D-A alternating TADF polymer and D-A orthogonal TADF polymer.

Nobuyasu et al. (2016) reported this type of TADF polymer for the first time. In their work, the electron donor was used as the main chain backbone, and the electron acceptor was introduced into the side chain to synthesize TADF emitter (PTZ-DBTO_2_) based on the phenothiazine donor and benzothiophene-s,s-dioxide acceptor. The donor and acceptor were covalently linked in a nearly vertical direction, creating a condition of Δ*E*_ST_ < 0.05 eV in zeonex. The device made of PTZ-DBTO_2_ shows an excellent performance, with an EQE of approximately 19%. Furthermore, they introduced dibenzothiophene unit into the backbone of the main chain, and then through copolymerizing with TADF small molecule, obtained a green light-emitting TADF polymer (COPO2) with strong conjugated structure. This COPO2 polymer emitted redshift, but had almost the same performance as the monomer PTZ-DBTO_2_. The OLED device based on COPO2 reached a maximum EQE of 11.05%. The research showed that the TADF performance of the designed COPO2 polymer depended on the performance of the PTZ-DBTO_2_ emitter core. To inhibit intramolecular and intermolecular exciton concentration quenching, Liu et al. (2018b) further copolymerized conjugated spacer units and TADF emitting monomers. Based on the above-mentioned TADF unit (PTZ-DBTO_2_), carbazole derivative was introduced into the main chain of the conjugated polymer. It was found that the content of the carbazole derivative unit could not only effectively suppress exciton quenching and non-radiative transition, but also control the distribution of molecular orbitals and Δ*E*_ST_ values, and could even adjust the properties of excited states. As the proportion of carbazole derivatives increased, the LUMO and HOMO energy levels of these TADF polymers increased, while the total energy gap and Δ*E*_ST_ decreased. Thus, three TADF polymers (HOMO, COP-50, COP-10) were synthesized by introducing different amounts of carbazole derivatives, wherein COP-10 showed a relatively high RISC rate and PLQY in film-state. Non-doped OLED devices based on COP-10 could achieve a maximum EQE of 15.7% at a lower turn-on voltage of 3.2 V and CIE coordinate of (0.46, 0.49).

In 2016, Cheng et al. (Zhu et al., 2016) proposed the concept of Backbone-donor/Pendant-acceptor and synthesized two alternative conjugated polymers PAPCC and PAPTC by improved Suzuki coupling copolymerization (see Figure 11). Among them, the donor was the commonly used wide bandgap carbazole and 9,10-dihydroacridine derivative unit, and a conjugate main chain having a high triplet level was obtained by 3,6-position copolymerization. The phenyl unit containing the electron-withdrawing group cyano or triazine was used as acceptor, which, as side chain, was chemically bonded to the N atom of 9,10-dihydroacridine that has a large dihedral angle to form pre-twisted intramolecular charge transfer structure. Time-density functional theory calculation indicated that in these two polymers, the HOMO delocalized over the entire backbone, while the LUMO located on the side of the acceptor. The high separation of HOMO and LUMO orbitals allowed the polymer to exhibit a relatively small Δ*E*_ST_ (PAPCC: 0.37 eV and PAPTC: 0.13 eV), achieving a maximum EQE of 12.6% in solution-processed PAPTC polymer OLEDs, with emission at 521 nm. Cheng's work provided evidence that the BDPA strategy could be used for the molecular design of new TADF polymers.

The article "Recent Advances in Thermally Activated Delayed Fluorescent Polymer—Molecular Designing Strategies" was published in 2020. Journal: Front Chem.

**Figure 11:** Chemical structure of the BDPA-type TADF polymer reported by the Cheng's team.

In order to further improve the EL performance of the device, Wang et al. (2018a) chose a more rigid acceptor, replacing tert-butyl group with benzene ring on the parent of triazine, and synthesized TADF emitting unit ATD [10-(4-(4-(4-6-diphenyl 1,3,5-triazine-2-) phenyl)−9,9-dimethyl-9,10-dihydroacridine]. By copolymerizing ATD-Br2 with two carbazole monomers, four conjugated polymers PCzATDx (x represents the molar content of ATD unit) were prepared. The experiments indicate that the TADF property of the small molecule ATD was completely retained in the polymer, showing a higher PLQY and a relatively small Δ*E*_ST_ value in the neat film. EL devices exhibited yellow emission with a maximum EQE of 15.5% and a PE of 50.5 lm W^−1^. More importantly, these devices exhibited low turn-on voltage of 2.53 V and low drive voltage of 4.05 V at 1,000 cd m^−2^ with a very low efficiency roll-off rate of only 0.5%, benefiting from the charge injection/transport in the polymer and the balance of the conjugate backbone.

To inhibit the intra- and inter-chain quenching process further, Cheng attempted to copolymerize TADF monomers with two carbazole monomers, and by adjusting the molar feed ratio, synthesized a series of conjugated polymers PCzAPTx with different TADF units (Zhu et al., 2018) (Figure 11). In these polymers, the carbazole oligomer, as a “block,” effectively regulated the distance between the TADF chromophores, suppressing the triplet quenching effect in the film. It has been found that the emission quenching process in polymers originated from intra- and inter-chain interactions between TADF chromophores, which depended to a large extent on the content of the APT TADF unit. By increasing the content of the carbazole block, PLQY increased from 50.0% (PCzAPT50) to 92.1% (PCzAPT10). The non-doped OLED device based on PCzAPT10 emitted yellow-green color, and had a maximum EQE of 16.9% and a low efficiency roll-off. Even at the brightness of 1,000 cd m^−2^, the EQE reached 15.6%, which was equivalent to 92.3% of the maximum EQE.

The article "Recent Advances in Thermally Activated Delayed Fluorescent Polymer—Molecular Designing Strategies" was published in 2020. Journal: Front Chem.

Despite this, the team members continuously synthesized a series of TADF conjugated polymer PABPC using the same carbazole/acridine donor as the backbone structure and the diphenyl ketone (BP) acceptor as the side chain pendant group (Yang et al., 2018a) (Figure 11). The TADF behavior was improved by controlling the content of ABP units in the polymer. In the pure film of PABPC5 with 5% mole content of ABP units, PLQY reached as high as 0.77. The best EL performance achieved in PABPC5-based device, such as a maximum EQE of 18.1% and a very slow efficiency roll-off with EQE of 17.8% at the brightness of 1,000 cd·m^−2^.

Based on the above-mentioned backbone structure, the team selected three isomers of benzoylpyridine derivatives with stronger electron-withdrawing ability than benzophenone as pendant acceptor groups, and regulated the side chain pendant unit to obtain long-wavelength emission. Three sets of corresponding conjugated polymers (PCzA3PyB, PCzAB2Py, and PCzAB3Py) were synthesized according to the BDPA strategy (Yang et al., 2019a). All polymers in the three series exhibited emission red-shift and distinct TADF characteristics, with a short microsecond delay lifetime (0.56 to 1.62 μs) and a small Δ*E*_ST_ (0.10–0.19 eV), compared to polymers with acceptor of dibenzophenone. Similarly, the different substitution patterns of pyridyl groups in the acceptor moiety also produced significant changes in PL properties. In PCzA3PyB, direct bonding of the pyridyl group to the main chain acridine unit resulted in a large red-shift of the polymer but a lower PLQY. On the contrary, distally linked pyridyl group separated by a benzoyl group caused a small red-shift but a higher PLQY in PCzAB3Py. In contrast, the preferred substitution of the pyridyl group is that the group is immobilized at the 2-position of the carbonyl group and located at the distal end of the acceptor moiety, forming a polymer with intramolecular hydrogen bonding and a phenyl linker, thereby synergistically providing a large red-shift and high PLQY. Using pure polymer film as the emitting layer in the corresponding device, PCzAB2Py5 showed better overall EL performance, with a maximum EQE of 11.9%, a low turn-on voltage of 3.0 V, and yellow light emission wavelength of 573 nm. It was worth mentioning that its efficiency roll-off rate was relatively low, with an EQE of 11.6% at the brightness of 1,000 cd·m^−2^.

The article "Recent Advances in Thermally Activated Delayed Fluorescent Polymer—Molecular Designing Strategies" was published in 2020. Journal: Front Chem.

Cheng's group (Wang et al., 2017) embedded the donor of TADF unit 2-(4-(diphenylamino)-phenyl)-9H-thioxanthone-9-9-10,10-dioxide (TT) into the main chain, and through copolymerizing with alternative fluorene and dibenzothiophene—s,s—dioxide fragments synthesized a series of BDPA TADF polymers (PFSOTTx). The twisted donor—acceptor structural units were covalently bonded to its donor fragment on the main chain, and the polymer had excellently inherited the characteristics of TADF small molecules used as monomers in copolymerization. By balancing the emission from the main chain and the TADF unit, the non-doped OLED exhibited white emission with CIE coordinate of (0.32, 0.31). According to the density functional theory calculations, HOMO mainly delocalized on the triphenylamine and fluorene segments, while LUMO localized on the side chain acceptor with a small overlap of HOMO-LUMO to ensure TADF characteristics. In addition, in a doped TADF polymer-based device with controlled TADF element content, the EQE with warm white emission was close to 10% and up to 19.4% with bright orange emission. One year later, they (Wang et al., 2018b) synthesized a series of BDPA-type conjugated polymers PCzDPTx composed of different contents of 3,6-carbazole and thioxanthone dioxide (DPT). It was found that the degree of conjugation increased with the increase of content of DPT unit in the PCzDPTx series polymer. The energy transfer between the carbazole fragment and the DPT unit occurred, and the emission peak gradually red-shifted. When the DPT content was 50%, PCzDPT50 polymer emitted red light. Similarly, the alternating copolymer PTD that contains 50% of DPT units emitted saturated red light. The doped PLEDs prepared based on the polymers PCzDPT50 and PTD produced saturated red electroluminescence, with CIE coordinates of (0.63, 0.37) and (0.64, 0.36), respectively. Clearly, it was feasible to control the emission color and improve the device EL performance by rationally designing and selecting suitable donors and acceptors, such as using long conjugated structures and rigid groups to suppress internal conversion rate through energy matching.

However, it is challenging to achieve a smaller Δ*E*_ST_ and a higher PLQY for orange to red TADF emitters due to high non-radiative internal conversion rates. Considering those problems, Xie and co-workers (Zhan et al., 2020) built, on their previous works, and selected a rigid anthraquinone group with the stronger electron-withdrawing ability to form a narrow bandgap TADF unit (TAQ). In comparison with fluorene group, the carbazole ring with stronger electron donating ability was introduced into the main chain, acting a better hole-transporting role. It was confirmed that the maximum emission peaks of the polymer PCzSOTAQx exhibited clear red shifts of 1–19 nm compared to PFSOTAQx. Impressively, the carbazole-based polymers PCzSOTAQx displayed better performances. This series of polymers showed higher PLQY (75%) and relatively smaller Δ*E*_ST_ values (0.12 eV) in the neat film. Especially, the OLED based on PCzSOTAQ2 achieved the saturated red emission with CIE coordinate of (0.62, 0.37) and a maximum EQE of 13.6%, which is the best one of the solution-processed OLEDs based on red TADF polymers reported so far. These results demonstrated that the red emission of conjugated polymer could be achieved simply by enhancing the strength of pendant acceptor and/or backbone donor, which supplied a useful guidance for the design and syntheses of efficient red-emitting TADF materials.

The article "Recent Advances in Thermally Activated Delayed Fluorescent Polymer—Molecular Designing Strategies" was published in 2020. Journal: Front Chem.

Friend's group (Freeman et al., 2017) designed a fully conjugated polymer ASFCN with donor and acceptor close to orthogonal configuration, which effectively eliminated the HOMO/LUMO overlap problem, making Δ*E*_ST_ small enough (<0.1 eV) to be overcome by heat and obtaining the TADF effect. They designed the synthesis of TADF polymers by using the acceptor as a side chain orthogonal to the donor backbone, which could greatly reduce the spatial overlap of the molecular frontier orbitals, ensure the conjugate along the polymer backbone, and retain the processability of the material and charge transport characteristics.

Park and Choi et al. (Kim et al., 2018) synthesized a green light-emitting TADF polymer P (DMAC-Cp) by introducing 1,1-diphenylcyclohexane (Cp) into the main chain of DMAC-TRZ. The introduced Cp not only acted as a linking group between the conjugated monomer units in the polymer emitter structure, breaking the conjugation along the polymer backbone, but also was conducive to regulating the solubility of the polymer. This novel polymer emitter possesses a very small Δ*E*_ST_ (0.023 eV) between the lowest singlet state and the triplet excited state. The TADF-OLED device, prepared by P(DMTRZ-Cp) polymer film emitter, exhibited a maximum EQE of up to 15.4% under green emission.

### Side Chain Type TADF Polymer

The main chain type TADF polymer is easy to form a large conjugated structure, while the synthesis is difficult due to the steric hindrance effect. Besides, those polymers have less advantage in the processing and preparation of the device for their inferior solubility and meltability.

The article "Recent Advances in Thermally Activated Delayed Fluorescent Polymer—Molecular Designing Strategies" was published in 2020. Journal: Front Chem.

In the side chain type TADF polymer, the TADF active unit is introduced as a pendant group into the conjugated or non-conjugated polymer backbone structure by chemical bonding. Due to the small conjugation effect of the polymer backbone, this type of TADF polymer supplies strategy to simply and efficiently achieve blue emission.

#### Conjugated Backbone

Yang et al. (Luo et al., 2016) first proposed a side chain engineering strategy for the development of TADF polymers in 2016, grafting active units with TADF behavior to the side chain positions of the polymer to achieve delayed emission. Since carbazole had a high triplet energy level and good hole transporting ability, it could be used as a main chain backbone of TADF polymer. When carbazole was grafted with different functional units (PXZ-OXD, TPA and Cz), a range of copolymers with different proportions of PXZ-OXD component, such as PCzn, could be synthesized through Suzuki copolycondensation. Among them, the polymer PCz12 showed the highest PLQY (33.7%). The PLED device prepared by this copolymer as a light-emitting layer had a maximum EQE of 4.3%, the peak EL wavelength of 506 nm, and the exciton utilization efficiency of 63.7%.

Xie et al. (2017) demonstrated in a further study that the side chain engineering strategy was an effective design concept for the synthesis of TADF polymers. Through Suzuki polycondensation of monomers M1, M2, and M3 under the feed molar ratio of 10:40:50, the authors obtained copolymer PCzDP-10 containing a high percentage of TADF components (72%), which exhibited up to 74% PLQY in an oxygen-free film state. By optimizing the device structure and energy transfer from the backbone to the TADF unit, the device based on the blue-green fluorescent polymer film achieved a maximum EQE of 16.1% at the brightness of approximately 100 cd·m^−2^, with CIE coordinate of (0.22, 0.40).

Based on the conjugated polymer, polyfluorene (see Figure 12), Yang et al. (2018b) regulated the conjugate length of the main chain by introducing 3,3'-dimethyldiphenyl ether on the backbone, and increased the triplet energy level of the main chain in the PFDMPE-based polymer from 2.16 to 2.58 eV to avoid the loss of triplet excitons. When red TADF emitter 2-(N-(4-oxooxyphenyl) diphenylamino)−4′-indole (ROC8) was further introduced as a side chain, an effective energy transfer from the host (PFDMPE) to the guest (ROC8) occurred in the solid state. The corresponding polymers (PFDMPE-R01 to PFDMPE-R10) exhibited distinct red TADF properties with a delayed fluorescence lifetime of 126–191 μs and a PLQY of 0.18–0.55. Among these polymers, PFDMPE-R05 exhibited the best device performance, with a bright red electroluminescence peak at 606 nm, and the current efficiency of 10.3 cd/A when EQE = 5.6%. However, the HOMO energy level of the host of fluorene and 3,3′-dimethyldiphenyl ether copolymer was 6.03 eV, which introduces a large hole injection barrier between the copolymer and the ITO anode modified by PEDOT:PSS, leading to a high device's turn-on voltage.

The article "Recent Advances in Thermally Activated Delayed Fluorescent Polymer—Molecular Designing Strategies" was published in 2020. Journal: Front Chem.

**Figure 12:** Chemical structures of side chain TADF polymers PFDMPE-R01 to PFDMPE-R10 and PCzDMPE-R03 ~ PCzDM PE-R10.

During immediate past, the group (Yang et al., 2019b) further selected carbazole that possesses a stronger electron donating ability instead of fluorene, designing and synthesizing red light TADF polymers (PCzDMPE-R03 ~ PCzDM PE-R10, see Figure 12) based on the main chains of carbazole and 3,3′-dimethyldiphenyl ether via Suzuki polycondensation. Compared with the red light TADF polymer based on the main chain of fluorene and 3,3'-dimethyldiphenyl ether copolymer, the new copolymers benefitted from the increase of the HOMO level of host and the improvement of hole injection ability. PCzDMPE-R07 showed the best performance of non-doped devices, including that the maximum current efficiency and EQE reached 3.35 cd/A and 2.03%, respectively, and the turn-on voltage was reduced from 9.8 to 5.2 V. In the optimized doping device, the current efficiency and EQE were further increased to 7.36 cd/A and 3.77%, respectively.

Zhou et al. (2019), inspired by the side chain engineering strategy for developing highly efficient TADF polymers, designed and synthesized a series of green TADF copolymers (Figure 13), which had different proportions of TADF units hanging on the side chains. To overcome the problem that the completely non-conjugated backbone was detrimental to charge transfer property and might result in poor device performance, in their work, the main backbone of the copolymer contained both a non-conjugated tetraphenylsilicon moiety and a conjugated carbazole unit in order to achieve equilibrium. Meanwhile, classical TADF unit 10,10′-(((2-(4-(9H-carbazol-9-yl) phenyl) pyrimidine−4,6-diyl) pyrimidine bis (4,1-phenylene) bis (10H-phenoxazine) (PXZ-Pm-MeOCz) was introduced as a side chain to impart TADF properties. All of these TADF polymers films exhibited high photoluminescence quantum yields in neat films, and when the TADF unit molar ratio in side chains was 6%, the PLQY reaches up to 71%. Using these polymers as the non-doped emissive layer, the solution processed PLED achieved fairly good performance, giving the maximum EQE of 7.0%, and CIE coordinate of (0.40, 0.54).

The article "Recent Advances in Thermally Activated Delayed Fluorescent Polymer—Molecular Designing Strategies" was published in 2020. Journal: Front Chem.

**Figure 13:** Chemical structure of side chain conjugated backbone TADF polymer.

#### Non-conjugated Backbone

Compared with the conjugated backbone TADF polymer, the non-conjugated skeletal TADF polymer has many advantages in synthesis simplicity and chemical modification. Moreover, the non-conjugated backbone has weak influence on the band structure of the TADF emissive unit, and is conducive to separately regulating the photoelectric performance of the TADF emitting unit.

##### Intramolecular charge transfer

By using phenothiazine as an electron donor and dibenzothiophene sulfone as an electron acceptor, Nobuyasu et al. (2016) synthesized a TADF small molecule. Then they obtained the TADF polymer through grafting the small-molecule TADF emissive unit and the TADF spacer unit benzene ring, as side chain, on the main chain of polyethylene, as shown in Figure 14. The maximum EQE of the PLED device prepared by this TADF polymer as the light-emitting layer was 2.3%. Subsequently, Bryce and Lee et al. (Li et al., 2017, 2018) prepared a series of TADF polymers by adjusting the ratio of dispersing units to TADF units in the polymer. It was found that the benzene ring in the side chain acted as a spacer unit which effectively prevents aggregation of the TADF unit and suppresses internal transition effect and TTA effect. With the increase of benzene ring content, the emitting efficiency of the polymer gradually enhanced, and simultaneously, the emission peak blue-shifted to some extent.

**Figure 14:** Side chain non-conjugated TADF polymers.

Lee et al. (Li et al., 2019a) developed a series of non-conjugated deep-blue TADF polymers based on polyethylene to produce highly efficient non-doped solution-processed PLEDs. In their designing strategy, an appropriate 9,9-dimethyl-10-phenylacridine (BDMAc) with high triplet energy (*E*_T_ = 3.38 eV) was incorporated as the host unit, which suppressed triplet energy from pendant emitter unit returning to the host, and thus prevented the device from performance deteriorating and promoted injection and transport of holes in the emitting layer. The deep-blue side chain pendant emitter had an extremely high PLQY of 90% and a suitable HOMO level (−5.50 eV), which is beneficial to synthesize polymers with unique TADF properties by adjusting the ratio of the bulk unit to the light-emitting unit. PLEDs based on these polymers as single emissive layers had a maximum EQE of 5.3%, an EL emission at 436 nm, and a CIE coordinate of (0.15, 0.09).

Park et al. (2019) used 9-vinylcarbazole (VCz) or 9,9-dimethyl-9,10-dihydroacridine as electron donors and phenyltriazine as electron acceptor, and synthesized the TADF emitting unit (VTD) by free radical copolymerization. By this way, they developed a highly efficient TADF PLED. In the polymer configuration, VCz and VTD monomers function as a host, and an emitter, respectively, and the copolymer composition that varies with the feed ratio of 9-vinylcarbazole and VTD affects the electroluminescent properties of the TADF PLED. It has been reported that when the feed ratio is 10%, the PLQY of the synthesized polymer is as high as 71%, and the PLED prepared by solution processing of the corresponding polymer achieved an EQE of 22.0%.

The article "Recent Advances in Thermally Activated Delayed Fluorescent Polymer—Molecular Designing Strategies" was published in 2020. Journal: Front Chem.

Besides common polyethylene, polynorbornene is also a good choice. It has a high triplet energy level (2.95 eV), which can effectively inhibit the reverse transfer of triplet from TADF units to the polymer backbone, and can be used to design blue light TADF polymers. Yang et al. (Zeng et al., 2018) introduced a hole injection unit, carbazole, and TADF small molecules into the norbornene polymer backbone as side chains, and synthesized a series of blue TADF polymers (PBD) by controlling the molar ratio of carbazole to TADF units (PBD-0, PBD-5, PBD-10, PBD-15, and PBD-20, Figure 14). As the proportion of TADF small molecule units increased, the degree of aggregation of the large conjugated structure led to a red-shift in the emission wavelength. The polymers all showed emission around 460 nm in pure films. By using these blue polymer emitters, the non-doped PLEDs produced achieved a maximum EQE of 7.3% and CIE coordinate of (0.20, 0.29).

##### Space charge transfer

The common system of intramolecular charge transfer is generally that the electron-donating group and the electron-withdrawing group are connected by a π-electron conjugated system. In the ground state, this system exhibits a polarization structure; and under photoexcitation, the dipole moment becomes intense and the Stokes shift increases, and thus, the charge transfer effect in the molecule enhances, and the emission of the molecule red-shifts. Therefore, the strong charge transfer effect in the conjugated structure generally causes a large red-shift in the emission wavelength of the TADF polymer, resulting in the orange-yellow and green-light emission in most of the TADF polymers. This is also the reason that the common intramolecular charge transfer system has been less used to the development of blue light TADF polymers. Recently, Shao and Wang broke through the design ideas of classic TADF materials with intramolecular charge transfer as the emitting mechanism, and put forward the design concept of “space charge transfer TADF polymer materials.” Combining aggregation-induced emission effect and TADF effect, they achieved PLED devices by solution processing of TADF polymer with the light emission coverage of deep-blue light (455 nm), red (616 nm) and the white.

The article "Recent Advances in Thermally Activated Delayed Fluorescent Polymer—Molecular Designing Strategies" was published in 2020. Journal: Front Chem.

Shao et al. (2017) first applied the space charge transfer concept to the design of TADF polymers, and proposed a new concept of blue TADF polymer design based on non-conjugated backbone and space charge transfer. The D and A units of this type of polymer were molecularly separated while spatially close, allowing a charge transfer process to occur through space rather than by binding to the acceptor, i.e., the space charge transfer effect occurs between the D and A units (Figure 15). A non-conjugated polyethylene was selected as the backbone, and a series of polymers having significant TADF characteristics were synthesized by free radical polymerization of the corresponding vinyl-functionalized acridone and triazine monomers. In this design strategy, the non-conjugated structure of the polymer avoided strong electron coupling between D and A, and was advantageous for controlling the charge transfer strength, thereby controlling the luminescent color. For example, in 95 mol% Ac and 5 mol% TRZ unit polymer, blue electroluminescence occurred with the CIE coordinate of (0.176, 0.269). Meanwhile, the spatial separation of D and A resulted in a small overlap of HOMO and LUMO, and thus Δ*E*_ST_ was very small (0.019 eV). Further, due to that the electron cloud of D and A was transmitted through spatial charge interaction, the spatial π-π interaction between D-A increased the rate of radiation transition. All these advantages impart the polymer fairly good luminescence properties, such as PLQY of 60% in the film state.

**Figure 15:** Chemical structures and molecular design of space charge transfer TADF polymers.

On the basis of previous studies, the research team further developed a general design strategy suitable for full-color TADF polymer (as shown in Figure 15) by regulating the charge transfer intensity between the donor and the acceptor (Hu et al., 2019). In the work, acridine was used as the electron donor and triazine as the electron acceptor, which was connected to the side chain of non-conjugated polystyrene. The space charge transfer intensity between the donor and different acceptors was regulated by using the substituent effect. The full-color emission of TADF polymer was realized, with a color region covering deep-blue (455 nm) to red (616 nm). In addition, by introducing two different donor/acceptor pairs (acridine/triazine pair and acridine/cyanotriazine pair to construct two space charge transfer channels) into the same polymer chain, the polymer emitted simultaneously blue and yellow light, achieving a white light emission. Their studies showed that the TADF polymers with space charge transfer had a small Δ*E*_ST_ (0.02 ~ 0.05 eV), and the HOMO / LUMO was effectively separated in space, leading to a typical TADF effect. Meanwhile, the aggregation induced emission effect was observed in the THF/H_2_O mixed solvent, and its emission intensity enhanced 117 times from solution state to aggregation state. It was found that the OLED devices based on the TSCT polymers of deep-blue, green, red and white light have good electroluminescent performance, with maximum EQEs of 7.1, 16.2, 1, and 14.1%, respectively.

The article "Recent Advances in Thermally Activated Delayed Fluorescent Polymer—Molecular Designing Strategies" was published in 2020. Journal: Front Chem.

### Self-Emission TADF Polymer

The synthesis of the above polymers deals with introducing a small molecular unit having TADF effect into the polymer. This conventional TADF polymer synthesis method, where the TADF small molecule itself is prepared in many steps and complicated in synthesis, with the addition of the other function groups, such as the solubilizing functional groups, polymerizable leaving groups, etc., makes preparation more difficult.

Wei et al. (2017) reported a method for achieving TADF properties in cyclic oligomers and polymers composed of non-TADF structural units. The research group, using an inductive conjugation idea, designed and prepared a simple repeating unit M1, with carbazole as the electron donor and benzophenone as the electron acceptor. Surprisingly, the individual light-emitting unit M1 exhibited only phosphorescence emission, but the Yamamoto-type polymer P1, obtained through polymerizing of M1, showed significant TADF behavior, with a PLQY up to 71%. It was explained that the polymerization of M1 extended the π-conjugated electron donor system, reducing the energy splitting between the corresponding ^1, 3^CT, making the Δ*E*_ST_ small (0.19 eV) enough to be overcome by heat while maintaining a sufficiently fast radiative decay rate. This study has fully demonstrated that a design strategy for TADF polymers could be developed by converting organic small molecules without TADF effect into high-efficiency TADF oligomers and polymers by induction binding.

Soon after, the team prepared a monochromatic OLED device based on the above self-emission TADF polymer P1 (Li et al., 2019b). They found that using P1 pure film or doping it in the host material, 1,3-bis9H-carbazol-9-ylbenzene (mCP), could realize cyan-blue light devices. The maximum EQE of the device with P1-doped mCP was 4.26%, while the EQE of the device based on P1 neat film was only 0.87%.

## Conclusion and Outlook

Theoretically, TADF materials have become the key technology for new OLEDs due to 100% exciton utilization. TADF materials and TADF-OLEDs have also made significant progress in recent years, especially small molecule TADF materials in achieving good performance of OLEDs with great success. Compared with TADF small molecule, TADF polymer performs better in preparing OLED devices with economical and efficient solution-process. However, unlike small molecule, TADF polymers have different molecular weights except dendritic macromolecules, and there are certain unavoidable defects in the structure, which makes the polymers not as easy to be optimized and repeated as small molecules. Now, TADF polymers still face many challenges, such as complex synthesis, limited variety, and relatively low efficiency of TADF-based devices. Compared with small molecules, most TADF polymers are only used as a carrier of TADF units, and cannot take advantage of the polymers' structural design preponderance. Therefore, it is expected that more and more TADF polymers not only have excellent processing properties, but also have advantages in synthesis, performance, and application.

The article "Recent Advances in Thermally Activated Delayed Fluorescent Polymer—Molecular Designing Strategies" was published in 2020. Journal: Front Chem.

### Synthesis

So far, some exciting results indicate that it is worthwhile to expand the corresponding research from small-molecule TADF emitters to TADF polymers emitters. However, it is undoubtedly challenging to obtain highly efficient and easily scalable TADF polymers due to synthetic limitations. Most of the existing TADF polymers are synthesized by embedding or grafting small-molecule TADF emitters into the polymer structure, which is not only limited by the variety of small-molecule TADF units, but also suffers from difficulties in complex polymerization methods, undefined structure and the possibility of unavoidable impurities. Thus, more attention is suggested to the three issues: simplification of synthesis method, reducing dependence on small molecules of TADF monomer, and understanding of structure-property relationships.

1. Simplification of synthesis method: Special attention should be paid to discovering simple synthesis methods, especially, finding the synthesis method to larger molecular structure and comonomer, and developing new synthetic strategies for preparing TADF polymers.
2. Reducing dependence on small molecules of TADF monomer: The development of TADF polymers is badly limited by the available small molecule active units, resulting in a limited number of TADF polymers. To change this situation, some specific polymer structures should be considered to achieve the TADF activity, reducing the dependence on small molecules of TADF monomer.
3. Understanding of structure-property relationships: More attention should be paid to complex interactions between donor and acceptor parts, polymer conjugation effects, charge transport and transfer effects, quenching effects, TADF monomer concentration effects, and intra- or intermolecular interactions of the TADF unit, rather than only optimizing the electronic state of the TADF emitting unit. Also, the effect of the content of the attachment sites and functional groups on the TADF polymer needs to be further studied.

The article "Recent Advances in Thermally Activated Delayed Fluorescent Polymer—Molecular Designing Strategies" was published in 2020. Journal: Front Chem.

### Property

Although TADF materials have made significant progress, TADF polymers still exhibit lower EQE values in both non-doped and doped devices than small molecule TADF devices. It is still difficult to obtain stable and efficient TADF polymer emitters and TADF-OLEDs with excellent performance for the following problems: (1) Generally, there is a contradiction between the separation of HOMO-LUMO orbitals and the suppression of IC process in TADF molecule. TADF polymers have a smaller Δ*E*_ST_ but relatively low quantum yields. (2) Embedding or grafting the active unit with TADF effect into the polymer structure is conducive to the delayed emission of the molecule. However, DF component depends on the exact position and content of TADF unit in the polymer, and negative effects such as exciton quenching may occur, increasing non-radiation decay. (3) Solution-processed polymer TADF devices suffer from more severe efficiency roll-offs, and at the same time, there are major problems with device stability and device efficiency. Therefore, the efforts are needed to solve the current problems of TADF polymers in OLED device applications and develop TADF polymers with better performance.

1. Development of TADF polymers with multiple luminous effects: (a) In aggregated state luminescent molecules, the ACQ makes the materials weaken in or even emit no fluorescence, which seriously affects the practical application of those materials. Therefore, it is necessary to find strategies to mitigate or eliminate the ACQ effect in polymers. Currently, the strategy of aggregation-induced emission or aggregation-enhanced emission molecular design was attempted to develop polymer light-emitting materials with AIDF effect, which is the most promising luminescent material for OLEDs and has great potential in the preparation of stable and efficient OLED devices. (b) More effective exciton utilization strategies are expected to be developed, in which materials not only emit thermally activated delayed fluorescence via reverse inter-system crossing from T_1_ to S_1_, but also emit room-temperature phosphorescence from the radiative decay of the lowest triplet state (T_1_) populated via IC process from the higher-lying triplet state (T_2_) or inter-system crossing from S_1_ to T_1_. These promising strategies may impart the new polymers long-life dual emission performance of delayed fluorescence and room temperature phosphorescence, while it is still a challenging research area.
2. Color purity of the TADF polymers: So far, almost all reported researches are concentrated in the green or orange-yellow TADF polymers, while blue and red corresponding TADF polymers are few, especially for deep-blue and pure blue. Those colors, however, are essential for full-color RGB displays. Therefore, new polymerization methods, geometric framework design and new construction groups should be explored, and more combination strategies should be developed to further optimize the displaying performance of TADF polymers.
3. Exploring stable host materials: Host materials are usually introduced into TADF polymers via chemical bonding for developing excellent non-doped TADF-OLEDs. In this case, the properties of host materials become very important, and new host materials, with good charge carrier transmission properties and good thermal and electrochemical stability, are still required to explore and develop.

The article "Recent Advances in Thermally Activated Delayed Fluorescent Polymer—Molecular Designing Strategies" was published in 2020. Journal: Front Chem.

### Applications

TADF-based materials are currently used in OLEDs, including (1) serving as host materials, guest materials and auxiliary dopants in doped OLED systems; (2) by mixing with phosphorescent materials or fluorescent groups to prepare white organic light-emitting diodes; (3) improving the efficiency of OLED devices with TADF molecular orientation; and (4) preparation of solution-processed OLEDs with better device performance.

Since TADF materials have the ability to utilize excitons by converting triplet excitons to singlet excitons, they are expected to be used in many other advanced fields, such as triplet-triplet annihilation sensitizers, electrochemiluminescence cells, organic ultraviolet photodetector, organic hybrid microelectronic radial heterojunction, light-emitting electrochemical cell, multicolor luminescent micelle, fluorescent probes and imaging, mechanoluminescence, and mechanoluminochromism. In all these applications, the small Δ*E*_ST_ of TADF materials and the effective RISC process in molecules are mainly utilized.

All in all, the research and development of TADF materials is still in the early stage. Besides the existing molecular systems, new TADF molecules should be explored. For this, new molecular design strategies and detailed theories should be established to construct materials with TADF characteristics and understand their photophysical properties.

## Author Contributions

All authors listed have made a substantial, direct and intellectual contribution to the work, and approved it for publication.

The article "Recent Advances in Thermally Activated Delayed Fluorescent Polymer—Molecular Designing Strategies" was published in 2020. Journal: Front Chem.

## Conflict of Interest

The authors declare that the research was conducted in the absence of any commercial or financial relationships that could be construed as a potential conflict of interest.
